The article "Analysis of Gut Microbiota in Patients with Exacerbated Symptoms of Schizophrenia following Therapy with Amisulpride: A Pilot Study" was published in 2022. Journal: Behav Neurol.

# Analysis of Gut Microbiota in Patients with Exacerbated Symptoms of Schizophrenia following Therapy with Amisulpride: A Pilot Study

**DOI:** 10.1155/2022/4262094

**Published:** 2022-03-05

**Authors:** Jinchi Zheng, Zeya Lin, Chih-Yuan Ko, Jian-Hua Xu, Yichuan Lin, Jinyi Wang

**Affiliations:** ^1^The Third Hospital of Quanzhou, Quanzhou, China 362000; ^2^Department of Clinical Nutrition, The Second Affiliated Hospital of Fujian Medical University, Quanzhou, China 362000; ^3^Department of Respiratory and Critical Care Medicine, The Second Affiliated Hospital of Fujian Medical University, Quanzhou, China 362000; ^4^School of Public Health, Fujian Medical University, Fuzhou, Fujian, China 350122; ^5^Respiratory Medicine Center of Fujian Province, Quanzhou, China 362000; ^6^Department of Tumor Surgery, The Second Affiliated Hospital of Fujian Medical University, Quanzhou, China 362000

## Abstract

Evidence is mounting that the gut microbiome is related to the underlying pathogenesis of schizophrenia. However, effects of amisulpride on gut microbiota are poorly defined. This study was aimed at analyzing cytokines and fecal microbiota in patients with exacerbated symptoms of schizophrenia treated with amisulpride during four weeks of their hospital stay. In the present study, feces collected from patients with schizophrenia were analyzed using 16S rRNA pyrosequencing and bioinformatic analyses to ascertain gut microbiome composition and fasting peripheral blood cytokines. We found that patients undergoing treatment of schizophrenia with amisulpride had distinct changes in gut microbial composition at the genus level, increased levels of short-chain fatty acid-producing bacteria (*Dorea* and *Butyricicoccus*), and reduced levels of pathogenic bacteria (*Actinomyces* and *Porphyromonas*), but the level of *Desulfovibrio* was still high. We also found a significant downregulation of butanoate metabolism based on functional analysis of the microbiome. After treatment, elevated levels of interleukin- (IL-) 4 and decreased levels of IL-6 were found. Our findings extend prior work and suggest a possible pharmacological mechanism of amisulpride treatment for schizophrenia, which acts via mediation of the gut microbiome.

## 1. Introduction

Schizophrenia (SCZ) is a psychiatric disease associated with psychosis, thought disorders, alterations in drive, volition, and neurocognition, affecting approximately 0.5% to 1.0% of the population worldwide, while the prevalence of SCZ is 5.44 per 1000 in China [1]. The developmental pathophysiological mechanism of SCZ is quite complex and has not yet been clearly elucidated.

Interestingly, shreds of evidence show that the gut microbiome may play a critical role in the pathogenesis of SCZ, and the pathophysiology involved in SCZ may also be regulated via the “microbiota-gut-brain” (MGB) axis [2, 3]. The composition of gut microbiota and its metabolites has been implicated in the development of SCZ. Alterations of bacterial taxa have been observed in SCZ, especially in decreased relative amounts of short-chain fatty acid- (SCFA-) producing bacteria and elevated pathogenic bacteria [4, 5]. Fecal microbiota transplantation techniques have been used to explore the mechanism of SCZ, including whether the gut microbiome of patients with SCZ modulates neurochemistry and neurologic functioning in rodents. These techniques demonstrated that the gut microbiome plays an important role in the development of SCZ [6, 7]. Additionally, gut-associated immune imbalances have also been demonstrated in patients with SCZ, particularly in relation to mucosal immunity [8], which is consistent with the developmental inflammatory hypothesis of explaining the pathogenesis of SCZ [9].

However, gut microbiota taxa are influenced by dietary habits, drugs, and environmental factors [10]. Our previous study revealed that antipsychotics can regulate metabolic and inflammatory abnormalities such as cytokines in patients with acutely exacerbated symptoms of schizophrenia [11]. Although drugs are a major therapeutic strategy for SCZ, many patients with SCZ have repeated episodes and experience medication side effects. A recent study found that olanzapine therapy in patients with SCZ altered gut microbiota including their metabolism [12]. However, the effect of amisulpride on gut microbiota has not been investigated in patients with schizophrenia, including whether the pharmacological mechanism of amisulpride treatment for SCZ acts via meditation of the gut microbiome.

Amisulpride is an effective, well-tolerated, and widely used dopamine D2 and D3 receptor antagonist for Chinese patients, which can improve SCZ symptoms effectively especially the negative symptoms of schizophrenia [13, 14]. Accordingly, we hypothesized that short-term therapy with amisulpride can ameliorate SCZ symptoms, mediated by the microbiome. The present study was aimed at investigating the microbiota composition of fecal samples as well as blood cytokines measured in a cohort of inpatients with SCZ who had acute exacerbated symptoms; the cohort's dietary intake and exposure to environmental factors were kept constant. The cohort was comprised of acutely exacerbated inpatients with SCZ, who were followed up for four weeks during amisulpride treatment.

## 2. Materials and Methods

### 2.1. Study Population

The Institutional Review Board of the Third Hospital of Quanzhou approved this study (IRB No. 2018001). All participants agreed to participate in this study and provided signed written informed consent before enrollment. Participants were recruited as inpatients at the Third Hospital of Quanzhou. The diagnosis of SCZ was based on Diagnostic and Statistical Manual of Mental Disorders (DSM) IV criteria. Participants were recruited when their symptoms were acutely exacerbated and treated with amisulpride (dosage from 400 to 1200 mg/kg) for 4 weeks during their hospitalization. Psychopathological status of the patients was assessed by senior physicians using the positive and negative syndrome scale (PANSS), consisting of positive, negative, and general psychopathology subscales.

Participants with the following characteristics were excluded from the study: unexplained first episode of SCZ; having been withdrawn from amisulpride treatment; having had amisulpride administered within the last 4 weeks; not having any follow-up blood and fecal samples; presence of infection, diarrhea, or gastrointestinal diseases; and having had antibiotics or probiotics administered within one month of recruitment. This study included 41 subjects. Five patients were excluded because they did not have follow-up blood or fecal samples, two because they had amisulpride administered less than 4 weeks ago, and one because he received another antipsychotic treatment, resulting in a final sample of 33 participants.

Participants received a standard hospital diet (i.e., 2000 ± 100 kcal, 55% ± 2% carbohydrates, 17% ± 2% protein, and 28% ± 2% fat per day), the same daily activities, psychoeducational activities, and occupational therapy. Fasting blood or fecal samples were collected following an acute episode admission on the following morning and then again the day before discharge in the morning.

### 2.2. Cytokine Analyses

Interleukin- (IL-) 1*β*, IL-4, IL-6, IL-10, tumor necrosis factor- (TNF-) *α*, and interferon- (IFN-) *γ* were assayed by BD Human Enhanced Sensitivity Cytometric Bead Array Kit (BD Biosciences, New Jersey, USA) as described previously [11].

### 2.3. Sampling, DNA Extraction, and 16S rRNA Gene Amplification Sequencing, Bioinformatic, and Predictive Function

All fresh fecal samples were collected and stored in a Microbiome Test Kit (G-BIO Biotech, Inc., Hangzhou, China). Total DNAs were extracted from fecal samples following the manufacturer's instructions. 16S rRNA sequencing was conducted as described for our previous study [15]. Based on the Quantitative Insights into Microbial Ecology bioinformatic pipeline for performing taxonomy assignments utilizing the operational taxonomic unit method, the total sequence data were used to analyze the fecal microbiota taxa. The Phylogenetic Investigation of Communities by Reconstruction of Unobserved States bioinformatic software package and the Kyoto Encyclopedia of Genes and Genomes (KEGG) were utilized to predict bacterial metabolic functions.

### 2.4. Statistical Analyses

Values are presented as the mean ± standard deviation. We analyzed differences in gut microbiota using the Wilcoxon signed rank sum test and performed principal coordinate analysis (PCoA) on the basis of the Bray–Curtis distance function, using R software (version 3.6.0). We performed chi-square and *t*-test analyses using the Statistical Program for the Social Sciences version 19.0 (SPSS Inc., Chicago, IL, USA). The significance level was set at 0.05.

## 3. Results

### 3.1. Participant Characteristics

Participants included 31 males and two females. After amisulpride treatment for 4 weeks, patients had lower diastolic blood pressure (*t* = 2.929, *P* < 0.005) and heart rate (*t* = 3.730, *P* < 0.001), but increased levels of triglyceride (*t* = −2.147, *P* = 0.036; Table 1). The follow-up data showed that IL-4 levels (*t* = −1.990, *P* = 0.050) were significantly increased and IL-6 levels (*t* = 2.039, *P* = 0.046) were decreased after amisulpride treatment (Table 1).

Using the PANSS, patients with schizophrenia with acutely exacerbated symptoms receiving amisulpride treatment for four weeks improved positive (*t* = 16.772, *P* < 0.001) and negative symptoms (*t* = 9.440, *P* < 0.001), general psychopathology (*t* = 16.475, *P* < 0.001), and total scores (*t* = 20.316, *P* < 0.001) (Table 2).

### 3.2. Characteristics of Sequencing Data

In terms of alpha diversity, we found that the difference in operational taxonomic units (OTUs) between amisulpride treatment before and after was not statistically significant (Figure 1(a)). After equalizing the library size to the minimum library size by random subtraction, we checked the average community diversity index (Chao (Figure 1(b)), Shannon (Figure 1(c)), and Simpson (Figure 1(d))) after equalizing library sizes to the minimum library size by random subtraction. We detected no statistically significant differences in community richness, diversity, and dissimilarity rank distribution (Figure 1(e)) before and after amisulpride treatment.

### 3.3. Alterations in Taxa Post Amisulpride Treatment

In terms of beta diversity, the gut microbiota before and after amisulpride treatment differed according to PCoA 1 and PCoA 2 (30.6% and 11.7%, respectively, Figure 2(a)). At the phylum level, we found no significant differences in relative amounts (data not shown). The relative amounts at the genus level were altered post amisulpride treatment in that *Dorea* (*P* = 0.031), *Desulfovibrio* (*P* = 0.045), and *Butyricicoccus* (*P* = 0.012) were increased, and *Actinomyces* (*P* = 0.042) and *Porphyromonas* (*P* = 0.045, Figure 2(d)) were decreased.

### 3.4. Predictive Functional Analysis

According to KEGG, the pathway of butanoate metabolism (*P* = 0.028) was significantly lower in the fecal microbiome post amisulpride treatment (Figure 2(e)).

## 4. Discussion

In this study, we found that inpatients treated with amisulpride for four weeks, showed elevated levels of IL-4 and decreased levels of IL-6. The relative amounts of genera in gut microbiome were altered. The genera of *Dorea*, *Desulfovibrio*, and *Butyricicoccus* were significantly increased; by contrast, *Actinomyces* and *Porphyromonas* were significantly decreased. The downregulation of butanoate metabolism was examined from functional analysis of microbiota post amisulpride treatment.

SCZ is a complex neurodevelopmental disorder. Growing and converging evidence from both genetic and environmental studies points to immune and inflammatory mechanisms as contributing a substantial risk for the development of this disorder [16]. Interestingly, the prevalence of psychiatric patients with irritable bowel syndrome has been found to be over 50% [17], and the estimated SCZ comorbidity with this disease approaches 20% [18]. Moreover, 50% of patients with SCZ have gastritis, 92% colitis, and 88% enteritis in an autopsy study [19]. The importance of inflammation and the involvement of the gastrointestinal tract in SCZ have received attention. The gastrointestinal tract is the human body's largest mucosal immune defense line and has abundant microbiota. Studies demonstrate that the gut microbial ecosystem has important links to host health, including cognition and behavior [3]. Neuroscience and microbiology have converged to begin to elucidate the role of microbes in brain development and function [3]. Microbes communicate with the brain via the MGB axis, encompassing the immune system and the production of microbial metabolites, such as SCFAs, which supports the hypothesis that the microbiome is related to SCZ [20, 21].

Intestinal symbiotic microorganisms can play a role in host immune regulation, while the disruption of gut permeability is initially a cascading factor; a decrease in SCFA production results in intestinal barrier dysfunction. However, SCFAs can maintain gut integrity, promote mucus synthesis, and reduce bacterial translocation [22, 23]. SCFAs primarily form from microbial fermentation of dietary fiber, including acetate, propionate, and butyrate. Additionally, SCFAs can regulate immune cells and play a vital role to maintain the balance of the intestinal immune microenvironment, have a direct anti-inflammatory effect on the intestine, and reduce the host's intestinal inflammatory response, which in turn reduces the release of TNF-*α*, IL-2, and IL-6 through the histone deacetylase inhibitory pathway [22, 23]. In the present study, acutely exacerbated SCZ inpatients treated with amisulpride showed increased SCFA-producing bacteria (*Dorea* and *Butyricicoccus*) and reduced pathogenic bacteria (*Actinomyces* and *Porphyromonas*).

Antipsychotics (phenothiazines and thioxanthenes) decrease gram-positive and gram-negative bacteria activity except amisulpride, which is a benzamide [24]. However, amisulpride is pharmacologically equivalent to sulpiride, and sulpiride has beneficial effects on gastrointestinal ulcers [25]. Interestingly, amisulpride significantly decreases levels of proinflammatory cytokines and elevates levels of anti-inflammatory cytokines [26, 27]. The decreased activity of immune factors (immunoglobulins, B lymphocytes, and HLA-DR^+^ cells) in patients undergoing SCZ treatment with amisulpride to balance the ratio of T-helper (Th)1/Th2 has been examined [28]. Moreover, amisulpride as a carrier combined with mesalazine, which is an anti-inflammatory drug, subsequently synthesizes to a new compound that could treat colonic diseases, and this new compound has an improved ability to decrease the levels of inducible nitric oxide synthase, cyclooxygenase-2, IL-1*β*, IL-6, and TNF-*α* [29]. Taken together, amisulpride has a potential anti-inflammatory effect. We speculate that amisulpride can regulate gut microbiota to achieve an anti-inflammatory effect.

Increasing SCFA-producing bacteria of acutely exacerbated SCZ inpatients is alleviated with amisulpride in this study. *Butyricicoccus* sp. was identified as a microorganism that could produce SCFAs [30]. Moreover, *Dorea formicigenerans* was enriched in SCZ; *Dorea* is part of the Lachnospiraceae family which can produce butyric acid [31]. Thus, it can be assumed to alleviate the inflammatory response and maintain intestinal epithelial function.

Nevertheless, large amounts of *Actinomyces* and *Porphyromonas* genera are observed in related inflammatory diseases. For example, large amounts of the *Actinomyces* genus have been identified in acute or remission SCZ patients [32]. By contrast, amisulpride treatment reduced these taxa in the current study. *Porphyromonas* sp. is a gram-negative and common periodontopathic bacterium, and we have reported large amounts of *Porphyromonas* spp. and elevated proinflammatory cytokines in patients with obstructive sleep apnea-associated hypertension [33]. Cooral administration of *Porphyromonas gingivalis* to intestine-induced diabetic mice has subsequently been found to lead to systemic inflammation and metabolic changes [34].

However, despite downregulation of butanoate metabolism analyzed from the microbiome, high levels of the pathogen *Desulfovibrio* were still present in this study, which is consistent with relevant literatures [4, 35]. *Desulfovibrio* is one of the mucin-degrading microbes, is a gram-negative bacterium, and is considered an opportunistic pathogen in the gut, as well as a potential lipopolysaccharide (LPS) producer [36, 37]. LPS causes mucin degradation, which disturbs the protection of gut mucosal surfaces and could potentially lead to a significant alteration in intestinal permeability, ultimately leading to bacterial translocation and intestinal leakage [38]. The increased circulating endotoxin levels then promote innate immunity events triggering low-grade systemic inflammatory processes, which may result in neurodevelopmental disorder [39]. Because butanoate metabolism of expression was decreased, we speculated a compensatory effect. In our previous study, where we investigated patients with schizophrenia with acutely exacerbated symptoms receiving antipsychotics, Th2 cytokine was markedly decreased in follow-up comparisons [11]. Another interpretation is that amisulpride has achieved the effect of reducing inflammation by increasing SCFA-producing bacteria and decreasing pathogenic bacteria, such that there was no need for excessive butyrate or other SCFAs. Another possibility is that production of reduced inflammatory metabolites from gut microbiota is not sufficient.

The main limitation of this longitudinal cohort study is the small sample size. Second, we did not compare the results between SCZ patients and healthy controls or patients receiving placebo. A prospective future study should be conducted with a larger sample size and healthy subjects to address this limitation. Third, we did not comprehensively analyze levels of endotoxins, SCFAs in blood/stool, or other immunity factors in the blood. Fourth, gut microbiota is perturbed by many factors, especially prehospitalization diet/environmental exposure such as alcohol use or smoking was unable to obtain accurate information from acute exacerbated patients. Fifth, microbiome fecal transplants researches [6, 7] are necessary to support our findings, and thus, caution is warranted when interpreting the pharmacological mechanism of amisulpride in SCZ related to the gut microbiome.

## 5. Conclusions

The present findings indicate distinct alterations of the fecal microbiome of acutely exacerbated SCZ inpatients during four weeks of treatment with amisulpride. Changes in the microbiome are associated with increased SCFA microbiota and reduced pathogen levels, as well as regulating the balance of cytokines but downregulating butanoate metabolism. This study provides some insights in the SCZ setting into the pharmacological mechanism of amisulpride in modifying the gut microbiome.

## Figures and Tables

**Figure 1:** Summary of sequencing data. Characteristics of sequencing data in the operational taxonomic units (OTUs) (a), the mean community diversity indices (Chao (b), Shannon (c), and Simpson (d)), and dissimilarity rank distribution (e). SCZ-AE: acute exacerbated schizophrenic patients; SCZ-T: treated with amisulpride for 4 weeks; ns indicates *P* > 0.05.

**Figure 2:** Gut microbiome composition at genus levels exhibits different patterns for acute patients with schizophrenia with acutely exacerbated symptoms (SCZ-AE) and those treated with amisulpride for 4 weeks (SCZ-T). Principal coordinate analysis (PCoA) based on the distance function of Bray–Curtis (a). Cladogram using LEfSe method showed the largest differences in taxa between SCZ-AE and SCZ-T (b). The color-coded bar chart shows the most prevalent genera present before and after in amisulpride treatment (c). Differences in the fecal microbiota at the genus level (d). Significant butanoate metabolism pathway downregulation was shown for the fecal microbiome in SCZ-T (e). Statistical analysis was performed with the Kruskal–Wallis test. ^∗^*P* < 0.05 compared with SCZ-AE.

**Table 1:** Changes of metabolic parameters and cytokines in amisulpride-treated patients. SCZ-AE: acute exacerbated schizophrenic patients; SCZ-T: SCZ-AE treated with amisulpride for 4 weeks; NA: not analyzed.

	SCZ-AE (*n* = 33)	SCZ-T (*n* = 33)	*t*-test/chi-square test	*P* value
Age (years)	38.5 ± 11.8	—	NA	NA
Height (cm)	170.7 ± 5.6	—	NA	NA
Body weight (kg)	67.4 ± 5.1	68.0 ± 5.1	-0.486	0.629
Systolic blood pressure (mmHg)	127.5 ± 12.0	126.9 ± 8.2	0.227	0.821
Diastolic blood pressure (mmHg)	83.4 ± 7.8	78.5 ± 5.3	2.929	0.0047
Heart rate (beats per minute)	83.8 ± 9.6	76.5 ± 5.5	3.730	0.00041
Fasting blood sugar (mmol/L)	5.7 ± 2.8	5.1 ± 2.6	0.997	0.322
Triglyceride (mmol/L)	1.2 ± 0.7	1.6 ± 0.8	-2.147	0.036
Total cholesterol (mmol/L)	4.4 ± 0.8	4.6 ± 0.8	-1.094	0.278
High-density lipoprotein cholesterol (mmol/L)	1.5 ± 0.4	1.6 ± 0.5	-1.316	0.193
Low-density lipoprotein cholesterol (mmol/L)	2.6 ± 0.8	2.6 ± 0.8	0.022	0.982
Interleukin-1*β* (pg/mL)	8.79 ± 6.74	7.14 ± 6.93	0.979	0.331
Interleukin-4 (pg/mL)	1.87 ± 0.82	2.53 ± 1.73	-1.990	0.050
Interleukin-6 (pg/mL)	6.83 ± 2.80	5.41 ± 2.86	2.039	0.046
Interferon-*γ* (pg/mL)	1.59 ± 0.31	1.72 ± 0.53	-1.243	0.218
Interleukin-10 (pg/mL)	0.67 ± 0.18	0.69 ± 0.30	-0.393	0.696
Tumor necrosis factor-*α* (pg/mL)	2.80 ± 0.48	2.56 ± 0.62	1.758	0.084

**Table 2:** Clinical disability measures. SCZ-AE: acute exacerbated schizophrenic patients; SCZ-T: SCZ-AE treated with amisulpride for 4 weeks.

PANSS subscales	SCZ-AE (*n* = 33)	SCZ-T (*n* = 33)	*t*-test/chi-square test	*P* value
Positive symptoms	24.1 ± 5.2	8.3 ± 1.7	16.772	<0.001
Negative symptoms	25.5 ± 6.3	13.5 ± 3.7	9.44	<0.001
General psychopathology	48.3 ± 5.6	27.3 ± 4.7	16.475	<0.001
Total scores	96.3 ± 11.5	49.8 ± 6.4	20.316	<0.001

## Data Availability

All the data used to support the findings of this study are included in the article.
